# How to Maintain a Sustainable Doctor-Patient Relationship in Healthcare in China: A Structural Equation Modeling Approach

**DOI:** 10.1155/2022/8251220

**Published:** 2022-07-05

**Authors:** Zhan-You Wang, Xin Zhang, Liang Ma

**Affiliations:** ^1^Management Science and Engineering, Shandong University of Finance and Economics, Jinan 250014, China; ^2^School of Labor and Employment Relation, Shandong Management University, Jinan 250014, China

## Abstract

It is important to identify means of improving and maintaining a sustainable doctor-patient relationship to address current healthcare issues. Although many studies have made outstanding contributions to the healthcare doctor-patient relationship literature, little work has been done to explore the influencing elements of the doctor-patient relationship in relation to expectation confirmation theory. To fill this gap, this study produced a theoretical framework model of the influencing factors of the doctor-patient relationship according to the expectation confirmation theory. Data from 335 Chinese patients were analyzed using a structural equation modeling method, and the results showed that patient satisfaction and patient trust are the most important factors in building a good relationship between doctor and patient. Furthermore, three components of postdiagnosis patient's perception, namely, perceived service quality, perceived communication quality, and perceived service attitude, are examined. These have a significant impact on patient confirmation. These three components ultimately affect the doctor-patient relationship. This study will be helpful for doctors to understand patients' service demands and their future diagnosis behavior. The proposals of this study may lead to optimization of the process of diagnosis and improvements in the quality of clinic services.

## 1. Introduction

It is important to improve the doctor-patient relationship in Chinese healthcare. The total number of medical damage liability disputes in 2020 was 18,670, an increase of about 3% over the number of cases in 2019 in China [1]. China has carried out many medical reforms, which have improved the quality of healthcare services. However, they play no role in tense doctor-patient relationships. For one thing, patients consider that cannot obtain benefits from appropriate services, and their interests may be harmed [2]. For their part, doctors hold that they face pressure from various social and economic aspects of healthcare while providing care [3]. Addressing the problem of improving the doctor-patient relationship in healthcare has become particularly urgent and necessary.

Scholars have made investigated the doctor-patient literature. Recent research focuses on patient's satisfaction, trust, and communication with doctors [4]; doctors' information system usage, attitudes, interpersonal skills, and description of treatment [5]; and the availability of particular skills, hospital equipment, and clinical capacity [6], among other topics. For example, Chandra et al. [7] found that mutual trust and communication were both positively correlated with patient satisfaction and perceived quality of healthcare services, leading to better adherence to medication regimes and following doctors' advice. Furthermore, Cheng et al. [8] showed that doctors' solicitude for their patients, their interpersonal communicative strategies, their discussion of the choice of treatment, technical skills, availability of medical supplies, and clinical competence jointly exert a significant and positive influence upon patient's satisfaction and the physician-patient relationship. Hu et al. [9] defined patient loyalty as willingness to repeat a treatment. If the healthcare service can retain patients and make them loyal customers, this will improve the doctor-patient relationship while also bringing long-term business benefits to hospitals. Naidu [10] identified that patients' perceptions, especially regarding doctors' communicative techniques, also significantly determine the degree of patient satisfaction. Although some studies have made outstanding contributions to the understanding of the doctor-patient relationship, few have explored how differences in perceived service quality affect the doctor-patient relationship and its process. Taking into account the important role of that different types of service quality have on the doctor-patient relationship [11, 12], unlike other studies, this study explores how different levels of perceived service quality affect the doctor-patient relationship. Clarifying this issue will be of great importance for understanding patient expectations and perceptions and improving a hospital's level of service quality [13].

Drawing on expectation-confirmation theory (ECT), this study proposed a research model to study how differences in perceived service quality of the patient affect the doctor-patient relationship and reveal its process. In this way, this study contributes to the doctor-patient relationship literature by examining how different levels of perceived service quality, such as perceived communication quality and perceived service attitude, and patient variables, such as the patient's expectation and patient's confirmation, affect the doctor-patient relationship, and reveal its process. Previous research emphasized the role of pre-existing factors of satisfaction while ignoring the mechanism of satisfaction emergence [10]. This study also contributes to the doctor-patient relationship literature with its use of ECT to identify how satisfaction is developed in the healthcare context. The practical contribution of this study is to allow hospital managers to fully understand the influence factors of doctor-patient relationship, thereby resulting in strategies to improve hospitals to retain patients. This study also expects that the results bring new insights to management in the medical services industry to further improve the operation performance of the medical service industry.

## 2. Theoretical Background

### 2.1. A Postacceptance Model of Expectation-Confirmation Theory

Oliver [14] proposed a postacceptance theoretical model in the form of ECT that consisted of five constructs, namely, expectation, perceived performance, confirmation, satisfaction, and continuance intention (repurchase intention). Here, expectation refers to an attitude that something should be in a certain way; early researchers defined expectations as the “beliefs that a given response will be followed by some event” [15]. In particular, expectation and perceived performance positively affected confirmation; expectation and confirmation positively affected satisfaction; and satisfaction prompted users' behavioral intention [13]. The postacceptance model of ECT has been generally accepted and extended across a variety of fields [16]. In addition, ECT-related studies, in most cases, added explanatory variables on the basis of the existing ECT to strengthen the explanatory power of the research or combined and compared with other theories to produce better verification results [17]. For example, Cheng [18] showed that the quality of information, system, supportive service, and instruction, to a large extent, contribute to perceived usefulness, confirmation, and flow, which jointly explain nurses' satisfaction with the application of blended E-learning system. On the basis of ECT, a group of researchers produced an integrated information system success model to study elementary parameters that affect consumers' continuous usage intention [19]. Delone and Mclean [20] have shown that system quality, information quality, and service quality all have a significant positive influence on users' confirmation, which further affects satisfaction. From the above discussion, this study posits that patient's expectation and different perceived service quality of patient, including service quality, communication quality, and service attitude positively influence patient's confirmation. Based on the above discussion and ECT, this study proposed the following hypotheses.

  H1: Patient expectation positively influences patient confirmation.
  H2: Perceived service quality positively influences patient confirmation.
  H3: Perceived communication quality positively influences patient confirmation.
  H4: Perceived service attitude positively influences patient confirmation.

A range of factors influence the degree of patient satisfaction in the context of healthcare sustainability. Lochman [21] identifies factors that are remarkably related to patient satisfaction, such as the accessibility of medical care, the organizational structure of clinics, treatment duration, doctors' ability to perceive, the clarity and retention of doctor-patient interactions, doctors' control, and patients' expectations. Amin and Nasharuddin [22] find that customer satisfaction conforms to customer expectations of products and services in relation to real performance. If the latter matches customers' expectations, they will be satisfied, and vice versa [23]. The ECT also postulates that the degree of satisfaction is generally determined by consumers' confirmation of expectations through premier usage, because consumers are used to comparing their expectations in the preliminary stage with the actual use experience. If their expectations are confirmed, they tend to be more satisfied with the systems or services [24]. Thus, this study holds that patients' expectations positively influence their satisfaction. Besides, according to ECT, when users are satisfied with specific services, they confirm the services, which means that their satisfaction positively influence patient's confirmation [25]. Lin et al. [26] also confirmed that satisfaction has a positive impact on customer confirmation. Based on the above discussion and ECT, this study proposes the following hypotheses.

  H5: Patient expectation positively influences patient satisfaction.
  H6: Patient satisfaction positively influences patient confirmation.

### 2.2. Relationship between Satisfaction and Doctor-Patient Relationship

In this study, patient satisfaction refers to a patient's emotional evaluation of a medical service by comparing their previous expectations with the service they actually received [27]. According to Naidu [10], patient satisfaction involves a variety of dimensions, including care quality, access, cost, physician's role and behavior, and physical facilities. On the other hand, patient satisfaction is a key factor in the establishment and maintenance of doctor-patient relationships in the provision of medical services [28]. Faezipour and Ferreira [29] indicated that an increase in patient satisfaction will also decrease the level of patient complaints; this, in turn, may significantly improve doctor-patient relationships. In addition, Garman et al. [30] found that patient satisfaction significantly increases patients' probability of returning to the previous provider for further treatment. In other words, patients' satisfaction with treatment gives rise to a positive relationship between the patient and the doctor, and appropriate and satisfying treatment of patients' results in lower levels of complaint and fewer medical disputes. Thus, improving patient satisfaction should be a key driver in improving doctor-patient relationships. Therefore, this study proposes the following hypotheses.

  H7: Patient satisfaction positively influences the doctor-patient relationship.

### 2.3. Relationship between Trust and Doctor-Patient Relationship

Trust is defined as a party's willingness to be vulnerable to the actions of another party based on the expectation that that other party will perform a particular action that is important to the trustor, irrespective of the ability to monitor or control that other party [31]. Given the credence product feature of healthcare services, patients must face uncertainties. Thus, trust matters in healthcare. In the online health services context, Mou et al. [24] confirmed that patients are more likely to perceive potential of benefits only if the online health information provider is trusted as reliable and competent. Kessler and Mylod [32] found a significant relationship between patient satisfaction and trust. Patient trust results in positive behavior, such as recommending medical services to relatives and friends, better compliance, and higher service use. An increase in the level of patient trust is likely to improve doctor-patient relationships because patients are more likely to visit again and recommend the doctor to others. In this study, if the patients complain less about the hospital and have more trust in its doctors, the doctor-patient relationship is thus greatly improved. From the foregoing, this study proposes the following hypotheses.

  H8: Patient satisfaction positively influences the patient's trust.
  H9: Patient trust positively influences the doctor-patient relationship.

Based on ECT, this study comes up with the research model shown in Figure 1. To measure different levels of service quality as perceived by patients, including perceived service quality, perceived communication quality, and perceived service attitude, this study also includes control variables, such as age, education, health status, cost to patient, and knowledge.

## 3. Materials and Methods

### 3.1. Variables and Measures

Questionnaires were used to validate the conceptual model (Table 1). All of the measured items were extracted from previously published studies: patient expectation was taken from Lin et al. [33]; perceived service quality, perceived communication quality, perceived service attitude, satisfaction, and trust were extracted from Fornell et al. [34]; confirmation was retrieved from Lin et al. [35]; and doctor-patient relationship improvement was adapted from Liang et al. [3]. The questionnaires included responses on a 5-point Likert scale.

### 3.2. Data Collection

This study provided the questionnaire through a survey platform (Soujump.com) that sent it to many WeChat groups and collected the answers. WeChat is the most popular social platform in China. WeChat had 1.21 billion users till November 2020. WeChat groups are created by WeChat users on the basis of similar interests or for specific purposes. A WeChat group is a group of people who can talk freely to other members in the group, which allows people with common interests to chat with each other. Everyone could be a member of different WeChat groups. Our participants were members from WeChat group.

The questionnaires were sent out from December 1 to December 8, 2020 to 3120 WeChat group users; 412 completed the survey, of which 77 were excluded for assessed inconsistencies. The remaining 335 valid questionnaires (81.3%) were used in this study. Basic respondent information is provided in Table 2.

### 3.3. Measurement Model

Structural equation modeling is a multivariate analytical method used to assess the consistency of hypothetical models and collected samples with reference to a theory [36–38]. This study adopted structural equation modeling to analyze the hypothetical model. Exploratory factor analysis and confirmatory factor analysis were carried out, followed by reliability and validity tests [39, 40]. The reliability and validity tests were performed using Cronbach's alpha, composite reliability, and average variance extracted (AVE) [41, 42]. The results provided in Table 3 indicate that the model had good reliability and validity. Cronbach's alpha was greater than 0.7, composite reliability was larger than 0.7, and AVE was greater than 0.5 [43]. The scale had good discriminant validity because the square root of the AVE of the measured variables was greater than their correlation coefficients [44]. The correlation coefficients are provided in Table 4, which shows that all measurement variables and potential variables had high correlation coefficients. However, the correlation coefficients of the other latent variables were low. This shows that the measurement items are internally consistent and possess good distinction capability [45].

## 4. Results

### 4.1. Results of Structural Model Analysis

The results of structural model analysis are shown in Figure 2. Patient expectation did not have a positive influence on confirmation (*β* = −0.002, *t* = 0.06); thus, H1 was not supported. Perceived service quality had a positive influence on confirmation (*β* = 0.320, *t* = 5.843), confirming H2. Perceived communication quality had a positive effect on confirmation (*β* = 0.145, *t* = 3.058), confirming H3. The impact of perceived service attitude on confirmation was significant (*β* = 0.478, *t* = 8.088), confirming H4. Patient expectation had a positive influence on satisfaction (*β* = 0.114, *t* = 3.040), confirming H5. Confirmation had a positive effect on satisfaction (*β* = 0.798, *t* = 25.346), confirming H6. Satisfaction had a positive influence on doctor-patient relationship improvement (*β* = 0.499, *t* = 8.556), confirming H7. Satisfaction had a positive effect on trust (*β* = 0.848, *t* = 45.227); thus, H8 was supported. Finally, trust had a positive effect on doctor-patient relationship improvement (*β* = 0.408, *t* = 6.607), confirming H9. From the results of the analysis of the control variables, this study found that serious disease has a positive effect on satisfaction (*β* = 0.077, *t* = 2.190). However, the influence of patient knowledge on patients' satisfaction is not significant (*β* = 0.036, *t* = 1.198).

### 4.2. Mediator Analysis

This study uses the bootstrap method as a test of the mediating influence of confirmation between perceived service quality and patient satisfaction, the mediating influence of patient satisfaction between patient confirmation and trust and between patient confirmation and doctor-patient relationship improvement, as well as the mediating influence of patient trust between patient satisfaction and doctor-patient relationship improvement. Specifically, this study uses the PROCESS SPSS macro developed by Hayes [46] to test mediation. The bias-corrected method and the percentile method are widely used to test the mediating influence, and the confidence level for the confidence intervals is 95%. The results are shown in Table 5.

Using the mediating influence criterion proposed by Prebensen and Xie [47], this study concludes that patient confirmation acts as a partial mediator between perceived service quality and patient satisfaction; patient confirmation acts as a partial mediator between perceived communication quality and patient satisfaction; and patient confirmation acts as a partial mediator between perceived service attitude and patient satisfaction. Thus, this implies that on the one hand, perceived service quality, perceived communication quality, and perceived service attitude have a positive influence on patient satisfaction; on the contrary, perceived service quality, perceived communication quality, and perceived service attitude affect patient satisfaction through patient confirmation. Furthermore, the results indicate that patient satisfaction acts as a partial mediator between patient confirmation and trust. This implies that on the one hand, patient confirmation has a positive influence on patient trust; however, patient confirmation affects patient trust through patient satisfaction. Further, patient satisfaction also acts as a partial mediator between patient confirmation and improvement in the doctor-patient relationship. This implies that on the one hand, patient confirmation has a positive effect on doctor-patient relationship improvement; on the other hand, patient confirmation affects doctor-patient relationship improvement through patient satisfaction. Finally, patients trust acts as a partial mediator between patient satisfaction and doctor-patient relationship improvement. This implies that on the one hand, patient satisfaction has a positive effect on doctor-patient relationship improvement; on the other hand, patient satisfaction affects doctor-patient relationship improvement through patient trust.

## 5. Conclusion

### 5.1. Key Findings

A summary of the research findings is presented in Table 6. First, our results show that patient expectation did not pay a positive role in confirmation with respect to the doctor-patient relationship. One possible explanation for this may be that confirmation is affected by the actual service level of hospital and doctors [48]. If the actual service level reaches the value expected by the patient, that patient will be confirmed; if the actual service level does not meet the expected value, the patient will not be confirmed [49]. Second, our results show that perceived service attitude has largest effect on patient confirmation, followed by perceived service quality and perceived communication quality. ECT suggests that performance has a positive effect on extent of confirmation [50]. This article takes the further step of dividing the performance part of the ECT framework into three dimensions, namely perceived service quality, perceived communication quality, and perceived service attitude, and it finds different intensities of influence on patient confirmation. Third, our results show that patient expectation and confirmation have a positive effect on satisfaction. This conclusion is also reached by Wu et al. [51] under the online impulse buying context. Fourth, patient satisfaction had a positive effect on trust, which further had a positive effect on doctor-patient relationship improvement. This kind of relationship is also proved by Liang et al. [4]. Finally, the mediator results show that patient confirmation acts as a partial mediator between perceived service quality and patient satisfaction, between perceived communication quality and patient satisfaction, and between perceived service attitude and patient satisfaction. Earlier work has shown that confirmation acts as a mediator between performance and satisfaction [52, 53]. This study takes the further step to find that patient satisfaction acts as a partial mediator between patient confirmation and trust and between patient confirmation and doctor-patient relationship improvement. Our results also showed that patient trust acts as a partial mediator between patient satisfaction and doctor-patient relationship. This relationship was also testified to by Zhang et al. [54].

### 5.2. Theoretical Implications

This study contributes to knowledge of the doctor-patient relationship by examining how patient-perceived levels of service quality affect the doctor-patient relationship and reveal its process. Although many studies have made outstanding contributions to the doctor-patient relationship literature [7, 8], few have explored the influencing factors of the doctor-patient relationship from different perceived service quality perspective. Considering that the doctor-patient relationship is basically affected by the difference between the patient's expectations and the actual service quality [1, 13]. Clarifying this issue is of great significance for understanding patient expectations and perceptions and improving the hospital's service quality levels [14]. Therefore, unlike other studies, this study applied the ECT to explain the influence mechanism of the doctor-patient relationship from the perspective of different perceived service quality. The results show that patient expectations did not have a positive effect on confirmation. However, perceived service quality, perceived communication quality, and perceived service attitude have a positive effect on confirmation, which further affects patient satisfaction, patient trust, and the doctor-patient relationship. This study expands the knowledge foundation of how patient expectation confirmation affects patient satisfaction, patient trust, and the doctor-patient relationship.

This study contributes to the sustainable doctor-patient relationships literature by identifying the mediator mechanism between patient perceived service quality and doctor-patient relationships. The literature on the doctor-patient relationship mainly focuses on patients' satisfaction, patient trust, and doctors' communication skills, information system usage, attitude, interpersonal skills, explanation of treatment, technical skills, hospital equipment, and clinical competence [55–57]. Unlike other studies, this study find that patient confirmation acts as a partial mediator between perceived service quality and patient satisfaction, between perceived communication quality and patient satisfaction, and between perceived service attitude and patient satisfaction. The results also showed that patient satisfaction acts as a partial mediator between patient confirmation and trust, patient confirmation, and the doctor-patient relationship. Finally, patient trust acts as a partial mediator between patient satisfaction and the doctor-patient relationship. This study expands the research framework of the doctor-patient relationship and enriches the research results about how patient expectation affects the doctor-patient relationship.

### 5.3. Practical Implications

This study has the following practical implications. First, according to our results, perceived service quality, communication quality and service attitude have a positive effect on patient confirmation, which further affect patient satisfaction, trust, and doctor-patient relationship improvement. Thus, for hospitals and doctors, it is wise to improve doctors' service quality, communication quality, and service attitudes because these can improve patient confirmation. Furthermore, the research results can provide a reference for hospital-level management, have practical guiding significance for doctor-patient crisis prevention, improve patient satisfaction, and enhance hospital brand image by improving communication methods and service attitudes in the process of consultation. Second, according to our results, patient confirmation positively affects patient satisfaction, which further influence patient trust and doctor-patient relationship improvement. Thus, for hospitals and doctors, it is wise to improve their service, and pay attention to patient confirmation because this will affect patient satisfaction, trust, and, ultimately, the doctor-patient relationship. Besides, through the discussion of the influencing factors of the doctor-patient relationship, it is possible to understand the patient's actual cognitive state of the doctor-patient relationship, which may serve as a good reference for follow-up research on improvements to the doctor-patient relationship. Finally, the ultimate goal of this article is to explore the influencing factors of the doctor-patient relationship and to call on researchers to foreground this doctor-patient relationship and ultimately establish a harmonious doctor-patient atmosphere.

### 5.4. Limitations and Future Research

Although this article makes a contribution to the research on the theoretical framework of the doctor-patient relationship, it results are constrained by the following research limitations: First, it may be limited by the research methods of questionnaire surveys, which produce subjective results, and there may be some deviations in the measurement [54]. Future research can use objective data to continue study of the research conclusions. Second, this article explores the factors that influence the doctor-patient relationship from the aspect of ECT and does not consider other potential factors, such as patient characteristics, doctor characteristics, or other similar factors. Future research should expand the theoretical model of influencing factors of the doctor-patient relationship proposed in this article. Finally, this article is a research conclusion drawn in the context of Chinese medical treatment and does not consider geographical differences among its respondents. Therefore, the research conclusions may have limited applicability. Future research can further verify the research conclusion in the Western context and discover potential differences between China and the West.

## Figures and Tables

**Figure 1:** Research model.

**Figure 2:** Results of structural model analysis.

**Table 1:** Questionnaire statements for usage factors.

Factors	Statements
Patient	I expect high-quality care before I go to the hospital
	I expect the medical services provided by the hospital to be very effective
Expectation (PE)	I expect medical care to be valuable compared to the price I pay

Perceived service quality (PSQ)	At present, you are satisfied with the treatment effect of your last visit
	Compared to the money you spent, you feel that the hospital's medical services are worth it
	Compared with the services you receive, you think the hospital's fees are reasonable

Perceived communication quality (PCQ)	The doctor can listen to you patiently and examine you carefully
	When the physician decides the treatment, he asks the patient (family member) for detailed advice
	The medical officer gives your consent prior to examination and treatment
	The medical staff offers you a variety of treatments

Perceived service attitude (PSA)	Doctors are easy to approach and friendly
	Doctors are highly skilled and trustworthy

Confirmation (CF)	The experience was better than I expected
	The level of service provided by the hospital was better than I had expected
	Most of my expectations for the hospital have been confirmed

Satisfaction (SF)	Generally speaking, this medical treatment process is satisfactory
	This medical treatment has reached your expectation of medical treatment
	Compared with other hospitals, I am satisfied with the service of this hospital

Trust (TR)	If I need to seek medical attention again, I prefer this hospital
	The possibility of you praising the hospital to others
	Your likelihood of recommending the hospital to someone else

Doctor-patient relationship improvement (DPR)	The doctor who treated me put me at ease
	The doctor who treated me was very concerned about me
	I complain less about hospitals
	I feel the doctor-patient relationship is less strained

**Table 2:** Respondents' basic information.

Demographic variables		Number	%
Gender	Male	116	34.63
	Female	219	65.37

Age	≤20 years old	32	9.55
	21–30 years old	67	20
	31–40 years old	131	39.10
	41–50 years old	90	26.87
	>50 years old	15	4.48

Education	Senior middle school or below	54	16.12
	Junior college	42	12.54
	Bachelor's degree	71	21.19
	Master's degree	128	38.21
	Doctor's degree or above	40	11.94

Income	<3,000	90	26.87
	3,000–4,999	43	12.83
	5,000–7,999	131	39.10
	8,000–11,999	55	16.42
	≥12000	16	4.78

Marital status	Unmarried	84	25.07
	Married	246	73.43
	Divorce	2	0.6
	Death of a spouse	3	0.9

Physical condition	Very good	85	25.37
	Relatively good	164	48.96
	General	77	22.98
	Relatively poor	8	2.39
	Very bad	1	0.3

Degree of illness at last visit	Very serious	0	0
	Relatively serious	13	3.88
	General	122	36.42
	Relatively mild	101	30.15
	Very mild	99	29.55

**Table 3:** Descriptive statistics and interconstruct correlations.

Items	Cronbach's alpha	CR	AVE	CF	DPR	PCQ	PE	PSA	PSQ	SF	TR
CF	0.925	0.952	0.869	0.932							
DPR	0.911	0.937	0.789	0.841	0.888						
PCQ	0.804	0.870	0.628	0.698	0.697	0.792					
PE	0.803	0.885	0.720	0.375	0.396	0.302	0.849				
PSA	0.833	0.923	0.856	0.806	0.808	0.728	0.379	0.925			
PSQ	0.850	0.909	0.770	0.745	0.714	0.642	0.475	0.696	0.878		
SF	0.923	0.951	0.866	0.854	0.845	0.691	0.422	0.771	0.782	0.931	
TR	0.939	0.961	0.892	0.798	0.831	0.621	0.352	0.724	0.691	0.848	0.944

Note: Patient expectation (PE); perceived service quality (PSQ); perceived communication quality (PCQ); perceived service attitude (PSA); confirmation (CF); satisfaction (SF); trust (TR); doctor patient relationship improvement (DPR).

**Table 4:** Cross loadings.

Items	CF	PCQ	PE	PSA	PSQ	SF	DPR	TR
CF1	**0.934**	0.647	0.320	0.762	0.705	0.781	0.766	0.739
CF2	**0.944**	0.690	0.355	0.762	0.717	0.823	0.811	0.784
CF3	**0.919**	0.615	0.373	0.730	0.661	0.783	0.774	0.708
PCQ1	0.659	**0.819**	0.295	0.699	0.619	0.652	0.644	0.579
PCQ2	0.604	**0.863**	0.306	0.599	0.577	0.597	0.628	0.521
PCQ3	0.408	**0.741**	0.119	0.438	0.420	0.440	0.421	0.391
PCQ4	0.489	**0.739**	0.190	0.523	0.368	0.454	0.465	0.438
PE1	0.305	0.251	**0.880**	0.304	0.371	0.337	0.320	0.252
PE2	0.367	0.295	**0.910**	0.360	0.443	0.426	0.390	0.357
PE3	0.271	0.214	**0.746**	0.294	0.392	0.294	0.287	0.277
PSA1	0.707	0.690	0.278	**0.918**	0.582	0.667	0.734	0.615
PSA2	0.782	0.660	0.416	**0.933**	0.700	0.755	0.761	0.720
PSQ1	0.636	0.577	0.422	0.610	**0.836**	0.693	0.626	0.583
PSQ2	0.685	0.557	0.428	0.613	**0.920**	0.710	0.636	0.616
PSQ3	0.639	0.558	0.401	0.610	**0.875**	0.654	0.617	0.620
SF1	0.812	0.668	0.360	0.727	0.764	**0.937**	0.778	0.771
SF2	0.810	0.635	0.420	0.750	0.749	**0.932**	0.781	0.772
SF3	0.762	0.628	0.397	0.675	0.669	**0.924**	0.801	0.824
TPR1	0.752	0.630	0.385	0.743	0.624	0.788	**0.905**	0.762
TPR2	0.745	0.588	0.353	0.718	0.605	0.697	**0.879**	0.711
TPR3	0.776	0.653	0.324	0.704	0.714	0.794	**0.900**	0.782
TPR4	0.713	0.604	0.347	0.708	0.587	0.719	**0.869**	0.693
TR1	0.708	0.560	0.303	0.643	0.613	0.785	0.737	**0.920**
TR2	0.788	0.595	0.353	0.723	0.657	0.804	0.812	**0.947**
TR3	0.764	0.603	0.341	0.684	0.686	0.814	0.805	**0.965**

**Table 5:** Results of mediating effects.

M/(IV)/(DV)	Items	Effect	Coefficient		Bias-coefficient percentile				Mediation existence
			SE	T	95% CI		95% CI		
CF/(PSQ)/(SF)	Direct effect	0.327	0.039	8.403	0.250	0.403	0.250	0.403	Partial
	Indirect effect	0.455	0.049	9.286	0.363	0.548	0.355	0.545	

CF/(PCQ)/(SF)	Direct effect	0.178	0.038	4.694	0.103	0.252	0.103	0.252	Partial
	Indirect effect	0.499	0.049	10.184	0.411	0.596	0.403	0.594	

CF/(PSA)/(SF)	Direct effect	0.232	0.046	5.011	0.141	0.323	0.141	0.323	Partial
	Indirect effect	0.536	0.053	10.113	0.434	0.639	0.431	0.638	

SF/(CF)/(TR)	Direct effect	0.273	0.054	5.066	0.167	0.379	0.167	0.379	Partial
	Indirect effect	0.525	0.054	9.722	0.424	0.627	0.417	0.624	

SF/(CF)/(DPR)	Direct effect	0.443	0.051	8.672	0.343	0.544	0.343	0.544	Partial
	Indirect effect	0.397	0.057	6.965	0.295	0.510	0.294	0.509	

TR/(SF)/(DPR)	Direct effect	0.498	0.051	9.783	0.398	0.598	0.398	0.598	Partial
	Indirect effect	0.346	0.053	6.528	0.237	0.442	0.243	0.446	

Note: Bootstrap 5000 times, IV: independent variable; M: mediator; DV: dependent variable.

**Table 6:** Summary of the research findings.

Hypotheses	Supported?
H1: Patient's expectations can positively influence patient's confirmation	No
H2: Perceived service quality can positively influence patient's confirmation	Yes
H3: Perceived communication quality can positively influence patient's confirmation	Yes
H4: Perceived service attitude can positively influence patient's confirmation	Yes
H5: Patient's expectation can positively influence patient's satisfaction	Yes
H6: Patient's satisfaction can positively influence patient's confirmation	Yes
H7: Patient's satisfaction can positively influence the doctor-patient relationship	Yes
H8: Patient's satisfaction can positively influence patient's trust	Yes
H9: Patient's trust can positively influence the doctor-patient relationship	Yes

## Data Availability

The underlying data supporting the results of this study can be accessed from the corresponding author.

## References

[1] Yi F. H. (2020). Big data report on national medical damage liability dispute cases. *Korean J Anesthesiol*.

[2] Hussain A., Sial M., Usman S., Hwang J., Jiang Y., Shafiq A. (2019). What factors affect patient satisfaction in public sector hospitals: evidence from an emerging economy. *International Journal of Environmental Research and Public Health*.

[3] Molina-Mula J., Gallo-Estrada J. (2020). Impact of nurse-patient relationship on quality of care and patient Autonomy in decision-making. *International Journal of Environmental Research and Public Health*.

[4] Liang C., Gu D., Tao F., Jain H. K., Zhao Y., Ding B. (2017). Influence of mechanism of patient-accessible hospital information system implementation on doctor-patient relationships: a service fairness perspective. *Information & Management*.

[5] Gong X., Zhang J., Siddiqui M. M. (2019). Effects of medical security satisfaction and trust in doctors on subjective well-being: evidence from China. *International Journal of Management and Sustainability*.

[6] Peng Y., Yin P., Deng Z., Wang R. (2019). Patient-physician interaction and trust in online health community: the role of perceived usefulness of health information and services. *International Journal of Environmental Research and Public Health*.

[7] Chandra S., Mohammadnezhad M., Ward P. (2018). Trust and communication in a doctor- patient relationship: a literature review. *Journal of Health Communication*.

[8] Cheng S.-H., Yang M. C., Chiang T. L. (2003). Patient satisfaction with and recommendation of a hospital: effects of interpersonal and technical aspects of hospital care. *International Journal for Quality in Health Care*.

[9] Hu H. Y., Chang H. C., Cheng C. C. (2016). Exploration on the relationship between patient satisfaction, relationship inertia and loyalty-switching barriers as the moderator. *Journal of Accounting Finance & Management Strategy*.

[10] Naidu A. (2009). Factors affecting patient satisfaction and healthcare quality. *International Journal of Health Care Quality Assurance*.

[11] Le W., Chang P.-Y., Chang Y.-W., Chen J. (2019). Why do patients move from online health platforms to hospitals? The perspectives of fairness theory and brand extension theory. *International Journal of Environmental Research and Public Health*.

[12] Grünloh C., Myreteg G., Cajander A., Rexhepi H. (2018). Why do they need to check me?” patient participation through eHealth and the doctor-patient relationship: qualitative study. *Journal of Medical Internet Research*.

[13] Guo S., Guo X., Zhang X., Vogel D. (2018). Doctor–patient relationship strength’s impact in an online healthcare community. *Information Technology for Development*.

[14] Oliver R. L. (1980). A cognitive model of the antecedents and consequences of satisfaction decisions. *Journal of Marketing Research*.

[15] Fishbein M., Ajzen I., Belief A. (1977). Belief, attitude, intention, and behavior: an introduction to theory and research. *Contemporary Sociology*.

[16] Hu M., Huang F., Hou H., Chen Y., Bulysheva L. (2016). Customized logistics service and online shoppers’ satisfaction: an empirical study. *Internet Research*.

[17] Lee Y., Kwon O. (2011). Intimacy, familiarity and continuance intention: an extended expectation-confirmation model in web-based services. *Electronic Commerce Research and Applications*.

[18] Cheng Y.-M. (2014). Extending the expectation-confirmation model with quality and flow to explore nurses’ continued blended e-learning intention. *Information Technology & People*.

[19] Pang S., Bao P., Hao W., Kim J., Gu W. (2020). Knowledge sharing platforms: an empirical study of the factors affecting continued use intention. *Sustainability*.

[20] Delone W. H., Mclean E. R. (2003). The DeLone and McLean model of information systems success:A ten-year update. *Journal of Management Information Systems*.

[21] Lochman J. E. (1983). Factors related to patients’ satisfaction with their medical care. *Journal of Community Health*.

[22] Amin M., Zahora Nasharuddin S. (2013). Hospital service quality and its effects on patient satisfaction and behavioural intention. *Clinical Governance: An International Journal*.

[23] Chakraborty R., Majumdar A. (2011). Measuring consumer satisfaction in health care sector: the applicability of servqual. *Researchers World*.

[24] Mou J., Shin D.-H., Cohen J. (2016). Understanding trust and perceived usefulness in the consumer acceptance of an e-service: a longitudinal investigation. *Behaviour & Information Technology*.

[25] Berry L. L., Bendapudi N. (2007). Health care. *Journal of Service Research*.

[26] Lin J., Wang B., Wang N., Lu Y. (2014). Understanding the evolution of consumer trust in mobile commerce: a longitudinal study. *Information Technology and Management*.

[27] Manzoor F., Wei L., Hussain A., Asif M., Shah S. I. A. (2019). Patient satisfaction with health care services; an application of physician’s behavior as a moderator. *International Journal of Environmental Research and Public Health*.

[28] Singh Gaur S., Xu Y., Quazi A., Nandi S. (2011). Relational impact of service providers’ interaction behavior in healthcare. *Managing Service Quality: International Journal*.

[29] Faezipour M., Ferreira S. (2013). A system dynamics perspective of patient satisfaction in healthcare. *Procedia Computer Science*.

[30] Garman A. N., Garcia J., Hargreaves M. (2004). Patient satisfaction as a predictor of return-to-provider behavior. *Quality Management in Health Care*.

[31] Mayer R. C., Davis J. H., Schoorman F. D. (1995). An integrative model of organizational trust. *Academy of Management Review*.

[32] Kessler D. P., Mylod D. (2011). Does patient satisfaction affect patient loyalty?. *International Journal of Health Care Quality Assurance*.

[33] Lin C.-P., Tsai Y. H., Chiu C.-K. (2009). Modeling customer loyalty from an integrative perspective of self-determination theory and expectation-confirmation theory. *Journal of Business and Psychology*.

[34] Fornell C., Johnson M. D., Anderson E. W., Cha J., Bryant B. E. (1996). The American customer satisfaction index: nature, purpose, and findings. *Journal of Marketing*.

[35] Lin C. S., Wu S., Tsai R. J. (2005). Integrating perceived playfulness into expectation-confirmation model for web portal context. *Information & Management*.

[36] Li X., Du J., Long H. (2020). Mechanism for green development behavior and performance of industrial enterprises (GDBP-IE) using partial least squares structural equation modeling (PLS-SEM). *International Journal of Environmental Research and Public Health*.

[37] Cho G., Hwang H., Sarstedt M., Ringle C. M., Sarstedt M., Ringle C. M. (2022). A prediction-oriented specification search algorithm for generalized structured component analysis. *Structural Equation Modeling: A Multidisciplinary Journal*.

[38] Collier J. E. (2020). *Applied Structural Equation Modeling Using AMOS: Basic to Advanced Techniques*.

[39] Alamer A., Marsh H. (2022). Exploratory structural equation modeling in second language research. *Studies in Second Language Acquisition*.

[40] Hasegawa Y., Lau S.-K. (2022). Comprehensive audio-visual environmental effects on residential soundscapes and satisfaction: partial least square structural equation modeling approach. *Landscape and Urban Planning*.

[41] Kursunoglu N., Onder S., Onder M. (2022). Evaluation of personal protective equipment usage habit of mining employees using structural equation modeling. *Safety and Health at Work*.

[42] Ringle C. M., Sarstedt M., Mitchell R., Gudergan S. P. (2018). Partial least squares structural equation modeling in HRM research. *International Journal of Human Resource Management*.

[43] Hair J. F., Black W. C., Babin B. J., Anderson R. E. (2009). *Multivariate Data Analysis*.

[44] Ma L., Zhang X., Ding X. (2020). Enterprise social media usage and knowledge hiding: a motivation theory perspective. *Journal of Knowledge Management*.

[45] Ma L., Zhang X., Ding X., Wang G. (2018). Bike sharing and users’ subjective well-being: an empirical study in China. *Transportation Research Part A: Policy and Practice*.

[46] Hayes A. F. (2013). Introduction to mediation, moderation, and conditional process analysis: a regression-based approach. *Journal of Educational Measurement*.

[47] Prebensen N. K., Xie J. (2017). Efficacy of co-creation and mastering on perceived value and satisfaction in tourists’ consumption. *Tourism Management*.

[48] Wang Y., Wu H., Lei X., Shen J., Feng Z. (2020). The influence of doctors’ online reputation on the sharing of outpatient experiences: empirical study. *Journal of Medical Internet Research*.

[49] Ccw A., Rh B., Wcb B., Jb C. (2020). Outsourcing success in the eye of the beholder: examining the impact of expectation confirmation theory on IT outsourcing - ScienceDirect. *Information & Management*.

[50] Park E. (2020). User acceptance of smart wearable devices: an expectation-confirmation model approach. *Telematics and Informatics*.

[51] Wu I.-L., Chiu M.-L., Chen K.-W. (2020). Defining the determinants of online impulse buying through a shopping process of integrating perceived risk, expectation-confirmation model, and flow theory issues. *International Journal of Information Management*.

[52] Mamun M. R. A., Senn W. D., Peak D. A., Prybutok V. R., Torres R. A. (2020). Emotional satisfaction and IS continuance behavior: reshaping the expectation-confirmation model. *International Journal of Human-Computer Interaction*.

[53] Nam K., Baker J., Ahmad N., Goo J. (2020). Determinants of writing positive and negative electronic word-of-mouth: empirical evidence for two types of expectation confirmation. *Decision Support Systems*.

[54] Zhang X., Ma L., Ma Y., Yang X. (2021). Mobile information systems usage and doctor-patient relationships: an empirical study in China. *Mobile Information Systems*.

[55] Cao Y., Zhang J., Ma L., Qin X., Li J. (2020). Examining user’s initial trust building in mobile online health community adopting. *International Journal of Environmental Research and Public Health*.

[56] Yan M., Tan H., Jia L., Akram U. (2020). The antecedents of poor doctor-patient relationship in mobile consultation: a perspective from computer-mediated communication. *International Journal of Environmental Research and Public Health*.

[57] Wang D., Liu C., Zhang X. (2020). Do physicians’ attitudes towards patient-centered communication promote physicians’ intention and behavior of involving patients in medical decisions?. *International Journal of Environmental Research and Public Health*.

